The article "Long non-coding RNA HOTAIR acts as a competing endogenous RNA to promote malignant melanoma progression by sponging miR-152-3p" was retracted in 2025. Reasons: manipulated images; duplicated images; original data or images not available.

# Long non-coding RNA HOTAIR acts as a competing endogenous RNA to promote malignant melanoma progression by sponging miR-152-3p

**DOI:** 10.18632/oncotarget.19910

**Published:** 2017-08-03

**Authors:** Wenkang Luan, Rubo Li, Liang Liu, Xin Ni, Yan Shi, Yun Xia, Jinlong Wang, Feng Lu, Bin Xu

**Affiliations:** ^1^ Department of Plastic Surgery, Affiliated People's Hospital of Jiangsu University, Zhenjiang, China; ^2^ Department of Neurosurgery, Affiliated People's Hospital of Jiangsu University, Zhenjiang, China; ^3^ Department of Neurosurgery, Nanjing First Hospital, Nanjing Medical University, Nanjing, China; ^4^ Department of Gastroenterology, Affiliated Hospital of Jiangsu University, Zhenjiang, China

**Keywords:** malignant melanoma, ceRNA, HOTAIR, miR-152-3p, c-MET

## Abstract

HOX transcript antisense RNA (HOTAIR) is associated with the growth and metastasis of many human tumors, but its biological roles in malignant melanoma remain unclear. In this study, we show that HOTAIR is overexpressed in melanoma tissues and cells, especially in metastatic melanoma. High HOTAIR levels correlate with poor prognosis in melanoma patients. We also determined that HOTAIR functions as a competing endogenous RNA (ceRNA) for miR-152-3p. miR-152-3p was decreased and acted as a tumor suppressor in melanoma, and c-MET was the functional target of miR-152-3p. Furthermore, HOTAIR promotes the growth and metastasis of melanoma cells by competitively binding miR-152-3p, which functionally liberates c-MET mRNA and results in the activation of the downstream PI3k/Akt/mTOR signaling pathway. We determined that HOTAIR acts as a ceRNA to promote malignant melanoma progression by sponging miR-152-3p. This finding elucidates a new mechanism for HOTAIR in melanoma development and provides a potential therapeutic target for melanoma patients.

## INTRODUCTION

Malignant melanoma, a cancer that originates from melanocytes, is the most aggressive type of skin tumor [1, 2]. The global incidence of malignant melanoma has been increasing in recent years [3, 4]. This type of tumor has a poor prognosis and is the primary cause of skin cancer-related death, mainly due to its metastatic phenotype and lack of efficient biomarkers [5]. The malignant progression of melanoma involves complex changes in networks of genes, signaling pathways and gene regulation [6, 7]. Hence, it is crucial to discover specific biomarkers and further explore the underlying molecular mechanisms of melanoma.

Non-coding RNAs (ncRNAs) are gene regulatory effector molecules, and their dysregulation contributes to the genesis and development of tumors, including melanoma [8–10]. Long non-coding RNAs (lncRNAs), a class of non-coding RNAs that exert critical effects in cancer biology, have recently been discovered [8, 11, 12]. The expression of lncRNAs could also be used as diagnostic or prognostic markers for numerous types of human tumors [13, 14]. Additionally, the aberrant expression of lncRNAs contributes to different biological processes in melanoma [15, 16]. Nevertheless, the role of only a few lncRNAs in the progression of melanoma have been identified.

The article "Long non-coding RNA HOTAIR acts as a competing endogenous RNA to promote malignant melanoma progression by sponging miR-152-3p" was retracted in 2025. Reasons: manipulated images; duplicated images; original data or images not available.

HOX transcript antisense RNA (HOTAIR) originates from the HOXC cluster and is the first lncRNA to be identified as being able to regulate gene expression [17]. Accumulating evidence has shown that HOTAIR promotes tumor cell invasion and metastasis in breast, pancreatic, and hepatocellular carcinomas [13, 18, 19]. HOTAIR may act as a competing endogenous RNA (ceRNA) in some types of cancer [20, 21], and is also associated with the motility and invasiveness of melanoma cells [22]. However, the molecular mechanism of the effect of HOTAIR in melanoma remains unclear. In this study, we showed that the expression of HOTAIR was increased in melanoma tissue and that HOTAIR overexpression was correlated with poor prognosis in melanoma patients. We also demonstrated that miR-152-3p functions as a tumor suppressor in melanoma by targeting c-MET. Furthermore, HOTAIR promoted the proliferation, invasion and migration of melanoma cells by acting as a ceRNA for miR-152-3p. The sponging of miR-152-3p by HOTAIR resulted in the loss of miR-152-3p suppression on the downstream target c-MET. In this way, HOTAIR affects melanoma progression by regulating the c-MET pathway. Thus, HOTAIR may serve as a survival indicator and potential therapeutic target for melanoma patients.

## RESULTS

### HOTAIR levels are elevated in melanoma and associated with poor prognosis in melanoma patients

We initially analyzed the HOTAIR expression in sixty malignant melanoma tissues and adjacent normal tissues by real-time PCR. HOTAIR expression was markedly increased in melanoma tissues compared to adjacent normal tissues (Figure 1A). In addition, HOTAIR levels were higher in metastatic melanoma tissues than in primary melanoma tissues (Figure 1B). Sixty melanoma patients were classified into two groups depending on their HOTAIR levels relative to the median ratio (2.96): the high HOTAIR expression group (n=30, HOTAIR expression ratio ≥ median ratio) and the low HOTAIR expression group (n=30, HOTAIR expression ratio < median ratio). As shown in Supplementary Table 1, high expression of HOTAIR was significantly associated with advanced clinical stage in melanoma, but not with age, sex, family history or ulcer. Kaplan-Meier analysis was used to evaluate the relationship between HOTAIR expression and overall survival of melanoma patients. The high HOTAIR expression group had a poorer survival rate than the low HOTAIR expression group (Figure 1C). We also detected HOTAIR levels in human melanoma cell lines (A375, A875, SK-MEL-1, SK-MEL-5 and SK-MEL-28) and human epidermal melanocytes (HEMa-LP and HEMn-LP) and found that HOTAIR expression was significantly higher in melanoma cells, especially in A375 and A875 cells (Figure 1D). These findings indicate that HOTAIR may contribute to the malignant progression of melanoma.

The article "Long non-coding RNA HOTAIR acts as a competing endogenous RNA to promote malignant melanoma progression by sponging miR-152-3p" was retracted in 2025. Reasons: manipulated images; duplicated images; original data or images not available.

**Figure 1:** HOTAIR levels are elevated in melanoma and association with poor prognosis of melanoma patients **(A)** HOTAIR levels were analyzed in sixty malignant melanoma tissues and adjacent normal tissues. **(B)** The level of HOTAIR was analyzed in primary melanoma tissues and metastatic melanoma tissues. **(C)** The overall survival curves of melanoma patients with high HOTAIR expression and low HOTAIR expression. **(D)** The HOTAIR expression profile in human melanoma cell lines (A375, A875, SK-MEL-1, SK-MEL-5 and SK-MEL-28) and human epidermal melanocytes (HEMa-LP and HEMn-LP). *P < 0.05, **P < 0.01, ***P<0.001.

### HOTAIR promotes the melanoma cell proliferation, invasion and migration and induces epithelial mesenchymal transition (EMT) *in vitro*

To further explore the biological function of HOTAIR in melanoma cells, we found that HOTAIR expression was significantly reduced by si-HOTAIR in A375 and A875 cells (Figure 2A). The CCK8 assay revealed that knockdown of HOTAIR significantly repressed the proliferative ability of A375 and A875 cells (Figure 2B and 2C). The colony formation assay confirmed the role of si-HOTAIR in inhibiting the proliferation of melanoma cells (Figure 2D and 2E). Subsequently, scratch wound assays and transwell assays showed that the migratory and invasive capacities of melanoma cells were inhibited by si-HOTAIR (Figure 2F–2I). Epithelial-to-mesenchymal transition (EMT) is as a crucial step during cancer cell metastasis [23]. Western blot was used to detect EMT marker expression. The expression of an epithelial cell marker (E-cadherin) was increased, whereas the mesenchymal marker (N-cadherin) was decreased in si-HOTAIR transfected melanoma cells (Figure 2J). This finding indicates that HOTAIR may promote melanoma cell invasion and migration by regulating EMT. Taken together, these results suggest that HOTAIR plays a significant role in promoting the growth and metastasis of melanoma.

**Figure 2:** The biological functions of HOTAIR in melanoma **(A)** Transfection efficiency of si-HOTAIR was determined by PCR. **(B** and **C)** The proliferative ability of A375 and A875 cells was measured by CCK8 assay after the cells were transfected with si-HOTAIR or NC. **(D** and **E)** The role of si-HOTAIR in inhibiting proliferation of melanoma cells was confirmed by colony formation assay. **(F** and **G)** The effect of si-HOTAIR on the migratory ability of melanoma cells was assessed by scratch wound assay. **(H** and **I)** The effect of si-HOTAIR on the invasive capacity of melanoma cells was assessed by transwell assay. **(J)** Western blot assays showed the levels of epithelial cell marker (E-cadherin) and the mesenchymal marker (N-cadherin) following transfection with si-HOTAIR or NC; GAPDH was used as a control. *P < 0.05, **P < 0.01, ***P<0.001.

The article "Long non-coding RNA HOTAIR acts as a competing endogenous RNA to promote malignant melanoma progression by sponging miR-152-3p" was retracted in 2025. Reasons: manipulated images; duplicated images; original data or images not available.

### Identification of miRNAs that bind to HOTAIR

Ahmad M. Khalil et al. have confirmed that HOTAIR is dual-localized lncRNAs (nuclear and cytoplasmic lncRNAs) by using FISH analysis [24]. We demonstrated this conclusion by using qRT-PCR of the preparation of cytoplasmic and nuclear fractions (Supplementary Figure 1E). Previous studies have shown that some specific lncRNAs may operate as competing endogenous RNAs (ceRNAs) in carcinogenesis. ceRNAs can function as miRNA sponges to modulate miRNAs, which functionally liberates mRNA transcripts targeted by miRNAs [25, 26]. We considered whether HOTAIR has the same effect in melanomagenesis. Starbase 2.0 (http://starbase.sysu.edu.cn/) was used to find miRNAs that potentially bind to HOTAIR, and 30 potential miRNAs that could interact with HOTAIR were predicted (Supplementary Table 2). To search for specific target miRNA of HOTAIR in melanoma, the miRNAs predicted above were measured by qRT-PCR in si-HOTAIR or NC transfected melanoma cells (Supplementary Table 3). miR-152-3p showed the highest upregulation after silencing HOTAIR in melanoma cells (Figure 3A). Furthermore, we detected the expression of miR-152-3p in melanoma tissues. miR-152-3p was downregulated in melanoma tissues compared to adjacent normal tissues (Figure 3B). The heat map data of sixty malignant melanoma tissues revealed the negative correlation between miR-152-3p and HOTAIR expression, and the Pearson correlation of HOTAIR and miR-152-3p levels was negative (Figure 3C and 3D). This negative correlation has also been proved in 51 melanoma tissues from TCGA database (Supplementary Figure 1A). Moreover, a miR-152-3p mimic decreased HOTAIR levels in melanoma cells (Figure 3E).

**Figure 3:** Identification of miRNAs that bind to HOTAIR **(A)** The expression levels of miR-152-3p in A375 and A875 cells following transfection with si-HOTAIR or NC. **(B)** miR-152-3p levels were analyzed in sixty malignant melanoma tissues and adjacent normal tissues. **(C)** The heat map shows that miR-152-3p is negatively correlated with HOTAIR in sixty malignant melanoma tissues. **(D)** The Pearson correlation of miR-152-3p and HOTAIR expression in sixty malignant melanoma tissues was negative. **(E)** The expression levels of HOTAIR in A375 and A875 cells following transfection with miR-152-3p mimic or NC. *P < 0.05, **P < 0.01, ***P<0.001.

The article "Long non-coding RNA HOTAIR acts as a competing endogenous RNA to promote malignant melanoma progression by sponging miR-152-3p" was retracted in 2025. Reasons: manipulated images; duplicated images; original data or images not available.

### HOTAIR directly binds to miR-152-3p

The potential miR-152-3p binding sites in HOTAIR transcripts were predicted using Starbase 2.0 (Figure 4A). We constructed luciferase reporter plasmids containing the wild-type HOTAIR (pMIR-HOTAIR-WT) and mutant HOTAIR with mutations in the predicted miR-152-3p binding sites (pMIR-HOTAIR-MUT). Dual luciferase reporter assays showed that a miR-152-3p mimic reduced the luciferase activity of pMIR-HOTAIR-WT but not that of pMIR-HOTAIR-MUT in melanoma cells (Figure 4B). miRNAs and siRNAs function through RNA Induced Silencing Complex (RISC), and Ago2 is an essential catalytic component of RISC that is involved in RNA cleavage [27–29]. We conducted a RNA immunoprecipitation (RIP) assay to explore whether HOTAIR functioned through the RISC complex via interaction with Ago2. In melanoma cells, RIP indicated that HOTAIR was preferentially enriched in Ago2-containing beads compared with the beads harboring control immunoglobulin G (IgG) antibody (Figure 4C and 4D). U1 small nuclear ribonucleoprotein (70 kDa, SNRNP70), a gene encoding the SNRNP70 protein associated with U1 spliceosomal RNA [30], was used as positive control. Moreover, we performed an RNA pull-down assay by using biotinylated miR-152-3p. HOTAIR was pulled down by biotin-labeled miR-152-3p oligos, but not the mutated oligos or biotinylated NC in melanoma cells (Figure 4E and 4F). These results suggest that HOTAIR directly binds to miR-152-3p in melanoma.

**Figure 4:** HOTAIR directly binds to miR-152-3p **(A)** The putative binding sites of miR-152-3p on the HOTAIR transcript, as predicted by starbase 2.0. **(B)** Over-expression of miR-152-3p led to a marked decrease in luciferase activity of pMIR-HOTAIR-WT, without any change in luciferase activity of pMIR-HOTAIR-MUT in melanoma cells. **(C** and **D)** Amount of HOTAIR bound to Ago2 or IgG measured by RT–qPCR after RIP. **(E** and **F)** Melanoma cells transfected with biotin-labeled miR-152-3p oligos (miR-152-3p-Bio) or mutated oligos (miR-152-3p-Bio-mut) or biotinylated NC (NC-Bio), assayed by biotin-based pull down after transfection. HOTAIR levels were analyzed by RT–qPCR. *P < 0.05, **P < 0.01, ***P<0.001.

### miR-152-3p represses melanoma cells proliferation, invasion and migration by targeting c-MET

miR-152-3p has been identified as a tumor suppressor gene in many human malignant tumors [31, 32]. It is essential to investigate the role of miR-152-3p in melanoma. As mentioned above, miR-152-3p expression was markedly decreased in melanoma (Figure 3C). We also detected the expression of miR-152-3p in human melanoma cell lines and human epidermal melanocytes. miR-152-3p was considerably lower in melanoma cells than in human epidermal melanocytes, especially in A375 and A875 cells (Figure 5A). The miR-152-3p mimic was transfected into A375 and A875 cells to further study the function of miR-152-3p in melanoma cells (Figure 5B). Overexpression of miR-152-3p suppressed the proliferation and the invasive and migratory abilities of melanoma cells (Figure 5C–5H). To study the mechanism of action of miR-152-3p in melanoma cells, we found that the binding sites of miR-152-3p matched the 3’-UTR of c-MET according to miRanda (http://www.microrna.org/) (Figure 5I). This suggests that c-MET is a potential target of miR-152-3p. c-MET acts as a oncogene in malignant melanoma, and c-MET expression was markedly increased in melanoma cells (Supplementary Figure 1D). The Pearson correlation of c-MET and miR-152-3p levels was negative in 51 melanoma tissues from TCGA database (Supplementary Figure 1B). Subsequently, we constructed luciferase reporter plasmids containing the wild-type (pMIR-c-MET-WT) and mutant (pMIR-c-MET-MUT) binding sites of the c-MET 3’-UTR. Dual luciferase reporter assays showed that over-expression of miR-152-3p led to a marked decrease in luciferase activity of the pMIR-c-MET-WT plasmid, while no significant changes were observed with the pMIR-c-MET-MUT plasmid in melanoma cells (Figure 5J). We also found that miR-152-3p up-regulation led to a decrease in the expression of endogenous c-MET mRNA and protein levels (Figure 5K and 5L), and the downstream PI3k/Akt/mTOR signaling pathway (Figure 5L). The effects of miR-152-3p on proliferation and the invasive and migratory abilities of melanoma cells were rescued by the c-MET plasmids (Figure 5C–5H, Figure 5K and L). Overall, we demonstrated that c-MET is a functional target of miR-152-3p in melanoma.

The article "Long non-coding RNA HOTAIR acts as a competing endogenous RNA to promote malignant melanoma progression by sponging miR-152-3p" was retracted in 2025. Reasons: manipulated images; duplicated images; original data or images not available.

**Figure 5:** c-MET is the functional target of miR-152-3p that affect proliferation, invasion and migration abilities of melanoma cells **(A)** The miR-152-3p expression profile in human melanoma cell lines (A375, A875, SK-MEL-1, SK-MEL-5 and SK-MEL-28) and human epidermal melanocytes (HEMa-LP and HEMn-LP). **(B)** Transfection efficiency of miR-152-3p mimic was determined by PCR. **(C** and **D)** Effect of miR-152-3p on the proliferative ability of melanoma cells was assessed by CCK-8 assay, c-MET plasmid reversed the effect of miR-152-3p. **(E** and **F)** The effect of miR-152-3p on the migratory ability of melanoma cells was assessed by the scratch wound assay, the effect of miR-152-3p was largely abrogated by the c-MET plasmid. **(G** and **H)** The effect of miR-152-3p on the invasive capacity of melanoma cells was assessed by transwell assay, and c-MET plasmid reversed this effect. **(I)** The binding sites of miR-152-3p within the 3′-UTR of c-MET were predicted by miRanda. **(J)** Overexpression of miR-152-3p suppressed luciferase activity in melanoma cells with the pMIR-c-MET-WT, but did not cause a significant change in melanoma cells with the pMIR-c-MET-MUT. **(K)** The expression of c-MET mRNA in melanoma cells transfected with miR-152-3p or miR-152-3p combination with the c-MET plasmid. **(L)** Western blots identifed c-MET protein expression and its downstream PI3k/Akt/mTOR signaling pathway changes following transfection with miR-152-3p alone or in combination with c-MET. *P < 0.05, **P < 0.01, ***P<0.001.

### HOTAIR acts as a ceRNA to promote melanoma cell growth and metastasis by sponging miR-152-3p

Because HOTAIR shares regulatory miR-152-3p with its target c-MET (Figures 4A and 5I), we further investigated whether HOTAIR acts as a sponge of miR-152-3p and promotes c-MET expression in melanoma cells. Dual luciferase reporter assays revealed that HOTAIR knockdown decreased the luciferase activity of pMIR-c-MET-WT, and the luciferase activity was rescued by miR-152-3p inhibitor in melanoma cells (Figure 6A). Moreover, knockdown of HOTAIR decreased the mRNA and protein levels of c-MET and the downstream PI3k/Akt/mTOR signaling pathway in melanoma cells (Figure 6B and 6C). However, this inhibition was attenuated by co-transfection of miR-152-3p inhibitor (Figure 6B and 6C). Importantly, the effect of si-HOTAIR on the proliferation, migration and invasion of melanoma cells was rescued by the miR-152-3p inhibitor (Figure 6D–6I). There was a positive correlation between HOTAIR and c-MET in 51 melanoma tissues from TCGA database (Supplementary Figure 1C). In summary, these results suggest an important role for HOTAIR in modulating the c-MET pathway by competitively binding miR-152-3p in melanoma.

**Figure 6:** HOTAIR promotes melanoma cell growth and metastasis by acting as a ceRNA **(A)** Luciferase activity of indicated groups in melanoma cells. **(B)** The expression of miR-152-3p and c-MET mRNA in melanoma cells transfected with si-HOTAIR or si-HOTAIR combination with miR-152-3p inhibitor. **(C)** Western blots identifed c-MET protein expression and its downstream PI3k/Akt/mTOR signaling pathway changes following transfection with si-HOTAIR or si-HOTAIR combination with miR-152-3p inhibitor. **(D** and **E)** miR-152-3p inhibitor reversed the effect of si-HOTAIR on the proliferative ability of melanoma cells. **(F** and **G)** miR-152-3p inhibitor reversed the effect of si-HOTAIR on the migratory ability of melanoma cells. **(H** and **I)** The effect of si-HOTAIR on the invasive ability of melanoma cells was largely abrogated by miR-152-3p inhibitor. *P < 0.05, **P < 0.01, ***P<0.001.

The article "Long non-coding RNA HOTAIR acts as a competing endogenous RNA to promote malignant melanoma progression by sponging miR-152-3p" was retracted in 2025. Reasons: manipulated images; duplicated images; original data or images not available.

### HOTAIR oncogenic activity functions in part through negative regulation of miR-152-3p *in vivo*

To further test the function of HOTAIR *in vivo*, we established a melanoma xenograft model by subcutaneously injecting A375 cells stably expressing control shRNA or shRNA-HOTAIR (Figure 7A). As shown in Figure 7B, the tumor volume in the control shRNA group was significantly greater than that in the shRNA-HOTAIR group between 15 and 30 days. After 30 days, the nude mice were sacrificed, and the tumor tissues were removed and weighed. The average tumor weight in the control group was significantly higher than that in the shRNA-HOTAIR group (Figure 7C). RT-PCR showed that the miR-152-3p levels were increased in the shRNA-HOTAIR group (Figure 7D). The expression of c-MET, Ki-67 (proliferation related) and N-cadherin (mesenchymal marker) was reduced, whereas the E-cadherin (epithelial cell marker) expression was increased in shRNA-HOTAIR group (Figure 7E). These results indicate that HOTAIR may promote melanoma growth and metastasis *in vivo* by operating as a ceRNA.

**Figure 7:** Inhibition of endogenous HOTAIR expression by shRNA inhibits melanoma growth *in vivo* **(A)** Tumor formation in nude mice and the excision tumor of A375 xenografts. **(B)** Difference in tumor volume between the NC group and the shRNA-HOTAIR group. **(C)** The tumor weight of excision tumor. **(D)** RT–qPCR identified miR-152-3p and HOTAIR expression changes. **(E)** The expression of c-MET, Ki-67, E-cadherin and N-cadherin was examined by Immunohistochemical staining of sections from melanoma xenograft model in nude mice. *P < 0.05, **P < 0.01, ***P<0.001.

## DISCUSSION

lncRNAs, non-coding RNAs longer than 200 nucleotides, have been implicated in a variety of cellular processes and critical functions related to cancer biology [33, 34]. The aberrant expression of lncRNAs may play a critical role in the occurrence and development of different tumors [35]. HOTAIR is significantly over-expressed in various types of cancer and promotes breast, pancreatic and hepatocellular carcinoma cell metastasis [13, 18, 19, 22]. We found that HOTAIR expression is also upregulated in melanoma tissues and cells, especially in metastatic melanoma. High HOTAIR levels correlate with poor prognosis of melanoma patients. Furthermore, we investigated the biological function of HOTAIR in melanoma cells. HOTAIR promotes melanoma cell proliferation, invasion and migration and induces EMT *in vitro*. Our data indicate that HOTAIR functions as an oncogene in melanoma. However, the molecular mechanism of HOTAIR in melanoma genesis and development remains unclear.

The article "Long non-coding RNA HOTAIR acts as a competing endogenous RNA to promote malignant melanoma progression by sponging miR-152-3p" was retracted in 2025. Reasons: manipulated images; duplicated images; original data or images not available.

In recent years, significant progress has been made in lncRNA research. Many studies have demonstrated that some specific endogenous lncRNAs can act as ceRNAs to interfere with miRNA pathways [25, 26]. The ceRNAs function as natural miRNA sponges that reduce the binding of endogenous miRNAs to their target genes, thereby regulating gene expression [36]. The disequilibrium of ceRNAs and miRNAs can be critical for tumorigenesis [37]. For example, the lncRNA Malat1 is overexpressed in gallbladder cancer and upregulates ANXA2 and KRAS by competitively binding to miR-206, thus promoting gallbladder cancer development [38]. Similarly, lncRNA Unigene56159 promotes epithelial-mesenchymal transition by acting as a ceRNA of miR-140-5p in hepatocellular carcinoma cells [39]. Additionally, HOTAIR promotes cancer progression by acting as a ceRNA. HOTAIR regulates HER2 expression by sponging miR-331-3p and promoting the proliferation, migration and invasion of gastric carcinoma cells [20]. Therefore, we hypothesized that HOTAIR may target miRNAs in melanoma.

To test this hypothesis, 30 potential miRNAs that could interact with HOTAIR were predicted using Starbase 2.0. The miRNAs predicted were measured by qRT-PCR after silencing HOTAIR in melanoma cells, and the results showed that miR-152-3p had the highest upregulation. On the other hand, overexpression of miR-152-3p suppressed HOTAIR expression, and the correlation between HOTAIR expression and miR-152-3p levels in melanoma tissues was negative. miRNAs function through the RNA-induced silencing complex (RISC), and Ago2 is an essential catalytic component of RISC [40]. Ago2 binds to miRNAs to promote their binding to mRNA, and in doing so participates in RNA silencing. We conducted a RIP assay to explore whether HOTAIR and miR-152-3p exist in the same RISC. Our results confirm that HOTAIR is enriched in Ago2-containing beads compared to controls. Dual luciferase reporter assays also confirmed that HOTAIR directly binds to miR-152-3p. Moreover, we performed an RNA pull-down assay by using biotin-labeled miR-152-3p oligos and found that miR-152-3p could pull down HOTAIR.

Accumulating evidence has shown that miR-152-3p is downregulated and functions as a tumor suppressor in many human tumors, including melanoma [41]. miR-152-3p promotes non-small cell lung cancer, colorectal cancer, and hepatocellular carcinoma cell growth and metastasis [31, 42, 43]. Here, we investigated the role of miR-152-3p in melanoma. miR-152-3p was largely reduced in melanoma and suppressed the proliferation, invasion and migration of melanoma cells. We also demonstrated that c-MET is a functional target of miR-152-3p. c-MET, a receptor for hepatocyte growth factor (HGF), contributes to tumor growth, EMT, invasiveness, and metastasis [44]. c-MET signaling promotes tumorigenicity in a variety of ways, including the highly oncogenic PI3K/AKT pathway [45]. c-MET has also been shown to be upregulated and function as an oncogene in melanoma [46, 47]. In addition, we found that knockdown of HOTAIR inhibits c-MET expression and the downstream signaling pathway PI3k/Akt/mTOR. This inhibition and the effect of HOTAIR on melanoma cells can be reversed by co-transfection of miR-152-3p inhibitor. These results reveal that HOTAIR promotes melanoma cell growth and metastasis by competitively binding miR-152-3p. Lastly, we demonstrated that HOTAIR promotes melanoma growth and metastasis *in vivo* through negative regulation of miR-152-3p.

The article "Long non-coding RNA HOTAIR acts as a competing endogenous RNA to promote malignant melanoma progression by sponging miR-152-3p" was retracted in 2025. Reasons: manipulated images; duplicated images; original data or images not available.

In conclusion, we demonstrated that HOTAIR is an oncogene in melanoma. HOTAIR promotes the growth and metastasis of melanoma cells by sponging miR-152-3p, functionally releasing c-MET mRNA transcripts targeted by miR-152-3p, and activating the downstream PI3k/Akt/mTOR signaling pathway. Understanding the regulatory mechanism of HOTAIR in melanoma could lead to the identification of novel therapeutic targets for melanoma. Future studies to assess the role of the HOTAIR/miR-152-3p/c-MET axis in a clinical context are warranted.

## MATERIALS AND METHODS

### Human tissues

A cohort of sixty malignant melanoma tissues (including 28 primary melanoma tissues and 32 metastatic melanoma tissues) and relative pair-matched adjacent normal tissues were collected from deferent melanoma patients who underwent surgical resection at The Affiliated People's Hospital of Jiangsu University. All the primary tumors were cutaneous melanomas and the metastatic melanoma tissues is lymph node metastases. The primary and metastatic lesions were derived from different patients. The clinical pathological features of the tissues of the patients were diagnosed by two pathologists, and no patients received chemotherapy or radiotherapy before surgery. The sample was stored in liquid nitrogen immediately after collection. The study was approved by the Human Research Ethics Committee of the Affiliated People's Hospital of Jiangsu University. Melanoma gene and miRNA expression data sets are were downloaded from The Cancer Genome Atlas (TCGA) data portal (https://cancergenome.nih.gov/).

The article "Long non-coding RNA HOTAIR acts as a competing endogenous RNA to promote malignant melanoma progression by sponging miR-152-3p" was retracted in 2025. Reasons: manipulated images; duplicated images; original data or images not available.

### Cell lines and cell culture

The human malignant melanoma cell lines A375 and A875 were purchased from The China Center for Type Culture Collection (Wuhan, China), and the human malignant melanoma cell lines SK-MEL-1, SK-MEL-5 and SK-MEL-28 were obtained by American Type Culture Collection (ATCC, USA). The cells were maintained in Dulbecco's modified Eagle's medium (Gibco, USA) supplemented with 10% fetal bovine serum (Invitrogen, USA) and antibiotics (100 μg/ml streptomycin and 100 U/ml penicillin). The human epidermal melanocytes HEMa-LP and HEMn-LP were purchased from Invitrogen (USA) and maintained in medium 254 and HMGS (Cascade Biologics). All cell lines were cultured in a humidified incubator containing 5% CO2 at 37°C.

### Oligonucleotides, plasmid construct and transfection

Oligonucleotides were chemically synthesized by GenePharma (Shanghai, China). The sequences were as follows: HOTAIR-small interfering RNA 1 (si-HOTAIR-1), 5′-GGAGAACACUUAAAUAAGUTT-3′; HOTAIR-small interfering RNA 2 (si-HOTAIR-2), 5′-AAAUCCAGAACCCUCUGACAUUUGC-3′; hsa-miR-152-3p mimic, 5′-UCAGUGCAUGACAGAACUUGG-3′; negative control (NC), 5′-UUCUCCGAACGUGUCACGUTT-3′. The short hairpin RNA (shRNA) was used to target HOTAIR, sense: 5′- CACCGCCTTTGCTTCGTGCTGATTCCGAAGAATCAGCACGAAGCAAAGGC -3′. The shRNA were synthesized and inserted into the pHBLV-U6 lentivirus core vector (Hanbio, Shanghai, China). For constructing HOTAIR plasmid, the full length of HOTAIR was amplified and inserted into pcDNA3.1 vectors (Invitrogen, USA). The pDONR223-MET plasmid was obtained from Addgene (USA). The oligonucleotides and constructs were transfected into melanoma cells using Lipofectamine 2000 reagent (Invitrogen, USA) according to the manufacturer’s instructions. The concentration of oligonucleotides and constructs were 100 nM and 250 ng/ul.

### RNA extraction and quantitative real-time PCR

Total RNA was extracted from cells and tissues using TRIZOL (Invitrogen, USA) according to the manufacturers’ instructions. We also separated nuclear and cytoplasmic fractions prior to RNA isolation by using a PARIS^™^ kit (Ambion) according to the manufacturer’s instructions. To detect the levels of miR-152-3p, HOTAIR and c-MET, reverse transcription (RT) was conducted with Fermentas reverse transcription reagents and an Applied Biosystems^®^ TaqMan^®^ MicroRNA Reverse Transcription Kit (Applied Biosystems, CA). The ABI StepOnePlus system (Applied Biosystems, CA) was used to perform the amplification reaction following predetermined conditions. The miR-152-3p primer was purchased from Guangzhou Ribo BioCoLTD (Guangzhou, China), U6 was used for normalization. For the analysis of the levels of HOTAIR and c-MET, GAPDH was used for normalization. GAPDH and U6 were used as reference in the cytoplasm and nuclear samples, respectively. The following primers were used: HOTAIR forward 5′-CAGTGGGGAACTCTGACTCG-3′ and HOTAIR reverse 5′-GTGCCTGGTGCTCTCTTACC-3′; c-MET forward 5′- CCCCACAATCATACTGCTGACA-3′ and c-MET reverse 5′-GTTGATGAACCGGTCCTTTACAG-3′; GAPDH forward 5′- GTCAACGGATTTGGTCTGTATT-3′ and GAPDH reverse 5′- AGTCTTCTGGGTGGCAGTGAT-3′. The 2^–∆∆Ct^ method was used to analyze the data.

The article "Long non-coding RNA HOTAIR acts as a competing endogenous RNA to promote malignant melanoma progression by sponging miR-152-3p" was retracted in 2025. Reasons: manipulated images; duplicated images; original data or images not available.

### Cell counting kit-8 (CCK-8) assay

CCK-8 (Beyotime, China) assay was applied to assess the proliferative ability of melanoma cells. We transfected the cells in the monolayer. After 24 hours of transfection, we detached and resuspended the cells for the desired assay. The transfected melanoma cells (5×10^3^ cells) were added to 96-well plates with 100 μl of culture media. At different times (12, 24, 36 and 48 h), the medium of each well was replaced with 100 μl fresh culture media contained 10% CCK8, and the cells were incubated for an additional 3 h at 37°C. The absorbance was measured using microplate reader (Multiscan FC, Thermo Scientific) at an optical density of 450 nm.

### Colony formation assay

We transfected the cells in the monolayer. After 24 hours of transfection, we detached and resuspended the cells for the desired assay. The transfected melanoma cells were seeded into six-well plate (100 cells/well). The cells were incubated for an additional 2 weeks, and were fixed with methanol and stained with 0.1% crystal violet. Visible colonies were manually counted.

### Cell invasion and migration assays

We transfected the cells in the monolayer. After 24 hours of transfection, we detached and resuspended the cells for the desired assay. Transwell assay was used to evaluate melanoma cell invasion ability. Transfected A375 cells were resuspended in serum-free DMEM and placed on the top of the Matrigel-coated invasion chambers (BD Biosciences, USA). 500 μl DMEM with 10% fetal bovine serum was added in the lower chamber. After 24 h, cotton swab was used to remove the non-invasive cells, and the invading cells were fixed and stained with 0.1% crystal violet. The cells were counted and photographed using a microscope (×100). We counted all the invading cells. Scratch wound assay was used to evaluate melanoma cell migration ability. Transfected A375 cells were seeded into 6-well plates, and 200 μl pipette tip was used to scratch the cell layers to form wound gaps. The cells were maintained in 10% FBS-supplemented DMEM. At 0 and 24 h, the cells were photographed an inverted microscope to record the wound width.

The article "Long non-coding RNA HOTAIR acts as a competing endogenous RNA to promote malignant melanoma progression by sponging miR-152-3p" was retracted in 2025. Reasons: manipulated images; duplicated images; original data or images not available.

### Western blot analysis

RIPA buffer (KenGEN, China) was used to extract the total protein from tissues and cells, and protein concentrations were quantified with BCA Protein Assay Kit (Beyotime, China). Equal amounts of protein were separated by 10% SDS-PAGE and transferred to PVDF membranes (Millipore, USA). Membranes were blocked with 5% nonfat milk and incubated overnight with diluted antibodies against c-MET (1:2000, Abcam, UK), PI3K (1:2000, Abcam, UK), pTyr458-PI3K (1:1000, CST, USA), AKT (1:1000, CST, USA), pSer473-Akt (1:1000, CST, USA), mTOR (1:1000, CST, USA), pSer2481-mTOR (1:1000, CST, USA), E-cadherin (1:1000, CST, USA), N-cadherin (1:1000, Abcam, UK), followed by incubation with HRP-conjugated secondary antibody (1:2500, Santa Cruz, USA). GAPDH was used as a control (1:2500, Abcam, UK).

### Luciferase reporter assay

The 3’-untranslated region (3’-UTR) fragment of c-MET containing the putative binding sequences of miR-152-3p were cloned into pMIR-REPORT vectors, and the fragment of HOTAIR including the binding site was inserted into pMIR-REPORT vectors. The mutated plasmid was used as the control. The melanoma cells were co-transfected with hsa-miR-152-3p mimic and related reporter constructs. The luciferase activity was detected using Dual Luciferase Reporter Assay System (Promega, USA) after transfection for 48 h.

### RNA immunoprecipitation (RIP)

RIP assay was performed using the EZ-Magna RIP™ RNA-Binding Protein Immunoprecipitation Kit (Millipore, USA). The melanoma cells were scraped off and lysed in complete RIP lysis buffer, and 100 μl of whole cell extract were incubated with RIP buffer containing magnetic beads conjugated with human anti-Ago2 antibody (Cell Signaling, USA). Positive control is SNRNP70 (Millipore, USA) and negative control is normal mouse IgG (Millipore, USA). PCR was used to detected the co-precipitated RNAs. Total RNAs (input controls) and IgG were also assayed to detecte whether the signals resulted from RNAs specifically binding to Ago2.

### RNA pull-down assay with biotinylated miRNA

Biotinylated miR-152-3p, biotinylated mutant miR-152-3p and biotinylated NC were synthesized by GenePharma (Shanghai, China), and were transfected into the melanoma cells using Lipofectamine 2000. The final concentration of each biotinylated miRNA was 20 nM. After 48 h, the cell lysates were incubated with M-280 streptaviden magnetic beads (Invitrogen, USA) as described previously [48]. The bound RNAs were purified using TRIZOL; RT–qPCR was used to detect the HOTAIR levels.

### Xenograft tumor assay

Ten immunodeficient female nude mice were used to test the effects of HOTAIR in malignant melanoma *in vivo*. Nude mice were obtained from Beijing Laboratory Animal Center (Beijing, China) and were divided into two groups (5 mice per group). A375 cells were transfected with shRNA or shRNA-HOTAIR lentivirus to establish a stabilized cell line. About 2×10^6^ logarithmically growing A375 cells stably expressing control shRNA or shRNA-HOTAIR were subcutaneously injected in nude mice, respectively. Tumor volume was measured every 5 days according to the formula (0.5 × length × width^2^). After 30 days, the nude mice were sacrificed and the tumor tissues were stripped and weighed. Total proteins and RNA were extracted from tissues, the expression of HOTAIR, miR-152-3p and c-MET were detected using western blot or qRT-PCR. The study was approved by the Experimental Animal Ethics Committee of the Affiliated People's Hospital of Jiangsu University.

The article "Long non-coding RNA HOTAIR acts as a competing endogenous RNA to promote malignant melanoma progression by sponging miR-152-3p" was retracted in 2025. Reasons: manipulated images; duplicated images; original data or images not available.

### Immunohistochemistry staining

Xenograft tumor sections were incubated with primary antibodies against c-MET (1:150, Abcam, UK), Ki-67 (1:100, Abcam, UK), E-cadherin (1:100, Abcam, UK), or N-cadherin (1:300, Abcam, UK) overnight at 4°C. Subsequently, the sections were incubated with a biotinylated secondary antibody (1:200, Gene Tech, China) at room temperature for 1 h. Then the sections were incubated with ABC-peroxidase for 1 h, staining with with diaminobenzidine for 5 min, counterstaining with hematoxylin (Gene Tech, China). Five randomly selected visual fields per section were assessed by 200 light microscopes to evaluate the effect of decreasing HOTAIR expression on the expression of c-MET, Ki-67, E-cadherin and N-cadherin. The percentage of positive tumor cells and the staining intensity were assessed.

### Statistical analysis

The data were presented as mean ±standard deviation (S.D.) and were analyzed with SPSS 13.0. T-test or one-way-ANOVA was used to measure the statistical significance of differences. Pearson correlation analysis was performed using MATLAB. Survival plots were generated by Kaplan-Meier analysis, log-rank tests were used to analyze the difference in overall survival time. P < 0.05 was considered to be statistically significant. All experiments were independently performed in triplicate.

## SUPPLEMENTARY MATERIALS FIGURE AND TABLES


